The article "Impact of Yiqi Huoxue Decoction on the Relationship between Remodeling of Cardiac Nerves and Macrophages after Myocardial Infarction in Rats" was retracted in 2023. Reasons: unreliable results or conclusions; concerns about the data; concerns about the peer review; concerns about the citations.

# Impact of Yiqi Huoxue Decoction on the Relationship between Remodeling of Cardiac Nerves and Macrophages after Myocardial Infarction in Rats

**DOI:** 10.1155/2022/4441603

**Published:** 2022-04-07

**Authors:** Yunke Liu, Shunwen Guo, Yuqin Zhang, Hui Wang, Jiani Wu, Wang'ou Lin, Binyue Zhang, Jie Chen, Yufei Li, Yunshu Zhang, Fanyu Wei, Tianhui Du

**Affiliations:** ^1^School of Traditional Chinese Medicine, Beijing University of Chinese Medicine, Beijing 100029, China; ^2^Fangshan Hospital Beijing University of Chinese Medicine, Beijing 102499, China; ^3^School of Acupuncture-Moxibustion and Tuina, Beijing University of Chinese Medicine, Beijing 100029, China; ^4^Wang Jing Hospital of CACMS, Beijing 100102, China; ^5^Yantai Puhui Hospital of Integrated Traditional Chinese and Western Medicine, Yantai 264004, Shandong, China; ^6^Guang'anmen Hospital China Academy of Chinese Medical Science, Beijing 100053, China

## Abstract

Sympathetic nerve remodeling after myocardial infarction (MI) has an indispensable role in cardiac remodeling. Numerous works have shown that sympathetic nerve remodeling can be delayed by inhibition of inflammatory response. Earlier studies have shown improvement in ventricular remodeling and inhibited chronic stage neural remodeling by Yiqi Huoxue decoction (YQHX). Therefore, the current study looked at the inhibitory effect of YQHX prescription on proinflammatory mediators and macrophages and the effect on neural remodeling at 3 and 7 days after MI. YQHX inhibited the expression of Toll-like receptor 4 (TLR4) and nuclear factor kappa B (NF-*κ*B) proteins and macrophage infiltration within 7 days after myocardial infarction. YQHX could decrease Th-positive nerve fiber density in the area around infarction and reduce the expression of growth-associated protein 43 (GAP43), nerve growth factor (NGF), and tyrosine hydroxylase (TH) proteins, which was associated with the remodeling of sympathetic nerves. Thus, the nerve remodeling inhibition after MI due to YQHX may be through its anti-inflammatory action. These data provide direct evidence for the potential application of traditional Chinese medicine (TCM) in the remodeling of sympathetic nerves after MI.

## 1. Introduction

In the past 20 years, MI (myocardial infarction) has been among the main causes of heart failure [1], and persistent arrhythmia after MI is also the main cause of sudden death [2]. In recent years, many investigations have demonstrated that sympathetic remodeling after MI is a crucial factor and the mode of triggering, initiating, and even maintaining malignant arrhythmias. Nerve repair and rearrangement occur in the infarcted area with the occurrence of ventricular remodeling after MI, which is called cardiac nerve remodeling. After MI, sympathetic nerves involved in cardiac innervation are damaged, and various local and circulating neurotrophic factors, for instance, GAP43 (growth-related protein 43) and NGF (nerve growth factor), participate in the repair process, resulting in excessive nerve sheath cells and axon regeneration around the infarcted tissue [3, 4]. Factors related to the remodeling of neurons play essential roles in reflecting sympathetic nerve function [5], promoting sympathetic nerve injury repair [6], and avoiding excessive growth [7]. However, cardiac remodeling is in a dynamic process, not a single repair or inhibition effect; it is also affected by a variety of factors, at different times or locations, or mutually promotes or antagonizes each other.

The article "Impact of Yiqi Huoxue Decoction on the Relationship between Remodeling of Cardiac Nerves and Macrophages after Myocardial Infarction in Rats" was retracted in 2023. Reasons: unreliable results or conclusions; concerns about the data; concerns about the peer review; concerns about the citations.

Increasing evidence indicates that the budding of a sympathetic nerve is closely associated with inflammation, mainly at the edge of infarction, where there are a large number of macrophages and inflammatory factors [8, 9]. Cytokines in the inflammatory environment can induce macrophage activation [10], thus promoting the expression of NGF [11], indicating that macrophages may also be involved in the regeneration and remodeling of sympathetic nerves. Wernli et al. [12] reported that chemical knockout of macrophages significantly reduces sympathetic nerve regeneration and NGF content after MI in rats. Hasan et al. [13] found that, after left ventricular myocardial tissue infarction in rats caused by left coronary artery ligation, sympathetic nerve remodeling and regeneration occur in the aggregation area harboring macrophages and fibroblasts. Through immunohistochemistry and in situ hybridization, NGF was found to be mainly synthesized and released by fibroblasts A and activated M-type macrophages, thus promoting sympathetic nerve remodeling. Macrophages generate a substantial count of proinflammatory cytokines and high levels of oxide metabolites, while M2 macrophages have an essential role in the repair of infarction by inhibiting destructive immune responses [14]. Anti-inflammatory treatment can reduce sympathetic remodeling after MI [15–17]. Thus, an anti-inflammatory drug is a promising approach for preventing sympathetic remodeling.

YQHX (Yiqi Huoxue decoction) is widely used to treat myocardial conditions considering its safety and efficacy. The formula comprises *Angelica Sinensis*, *Astragalus membranaceus*, *ginseng*, *Ligusticum chuanxiong*, and *Panax notoginseng*. According to the qi and blood theory of traditional Chinese medicine, YQHX can nourish the heart and qi, promote blood circulation, and clear veins. YQHX has been shown to improve ventricular remodeling in rats [18], improve mitochondrial function [19], regulate energy metabolism [20, 21], block the expressions of neural remodeling factor and cardiac hypertrophy protein within the chronic stage, and reduce cardiac hypertrophy and nerve remodeling [22], to achieve the effect of alleviating MI injury.

The article "Impact of Yiqi Huoxue Decoction on the Relationship between Remodeling of Cardiac Nerves and Macrophages after Myocardial Infarction in Rats" was retracted in 2023. Reasons: unreliable results or conclusions; concerns about the data; concerns about the peer review; concerns about the citations.

Although YQHX can reduce nerve remodeling, whether it can improve sympathetic remodeling of the heart by regulating the phenotypic transformation of macrophages needs more research. Hence, in the current work, the function of macrophages in sympathetic remodeling after MI was evaluated, and the potential of YQHX to inhibit sympathetic remodeling after MI was determined by regulating the differentiation of macrophages.

## 2. Reagents and Methods

### 2.1. Ethical Approval

The current study was approved by the Medical and Laboratory Animal Ethics Committee, Beijing University of Chinese Medicine (ETHICS No.: BUCM-4-2018071701-3002). All the animal studies were carried out following the National Institutes of Health Guidelines for the Care and Use of Laboratory Animals (NIH Publication No. 85-23 and revised in 1996) guidelines.

### 2.2. Herb Preparation

YQHX comprises five herbs: *Angelica sinensis*, *Astragalus membranaceus*, *Ligusticumchuanxiong Hort*, *Panax ginseng* C. A. Meyer, and *Panax notoginseng*. Each of these herbs was procured from Dongzhimen Hospital, Beijing University of Chinese Medicine. The high-performance liquid chromatography coupled with linear ion trap quadrupole Orbitrap high-resolution mass spectrometry (HPLC-LTQ-Orbitrap MS) method was applied with DDA-MS2 information acquisition and earlier studies for examining the components of YQHX aqueous extracts systematically, and 87 compounds were inferred, in addition to the structural types of flavonoids and triterpenoid saponins, including panaxosides, ginsenosides, floralginsenoside, astragaloside, and quinquenoside. As per the recommended active pharmaceutical ingredients (API) dose for the human body (of 96 g/d), the rat dose was six times the relative dose ratio for the human body. Hence, a drug dose equal to 8.2 g/kg was selected; earlier studies have furnished sufficient evidence for the effectiveness of this dose [19].

### 2.3. Animal Model Establishment and Group Administration

Adult male specific-pathogen free (SPF) Sprague Dawley (SD) rats (200 ± 20 g) were procured from Beijing Weitong Lihua Laboratory Animal Science and Technology Co., Ltd. (Certificate Number: SCXK2016-0006). Adaptive feeding for three days before MI surgery was performed in the Animal Experimental Center, Beijing University of Chinese Medicine. In the period for feeding, the rats were freely provided with distilled water and a regular diet. A constant humidity and temperature were maintained in the laboratory. An earlier published method was followed to establish the rat MI model [23]. Experimental surgery was performed aseptically with pentobarbital sodium (1%, 40 mg/kg) for abdominal anesthesia. Postendotracheal intubation, an animal ventilator of small size, was connected (breathing rate of 85 times/min) at a breathing ratio of 1 : 2. To make the model, ligation of the descending anterior branch of the left coronary artery was performed through 5-0 nylon suture, and the thoracic cavity was closed layerwise. The same procedure was performed on the control rats except for left anterior descending (LAD) ligation. The significant elevation of the ST segment under electrocardiogram (ECG) limb lead monitoring confirmed the successful modeling of MI (Shanghai Medical Electronic Instrument Factory).

The article "Impact of Yiqi Huoxue Decoction on the Relationship between Remodeling of Cardiac Nerves and Macrophages after Myocardial Infarction in Rats" was retracted in 2023. Reasons: unreliable results or conclusions; concerns about the data; concerns about the peer review; concerns about the citations.

The rats were arbitrarily categorized into the sham operation group (*n* = 10) and the infarction group (*n* = 10). In the infarction group, ECG examination was carried out on day 2 after operation, and more than four Q-wave numbers met the requirements of the experiment. Rats having identical Q-wave numbers were arbitrarily categorized into two groups. Ten rats without ligature were selected as the sham operation group. SD rats with successful ligation were arbitrarily categorized into three groups: the MI model (MI, *N* = 10), the MI model + invigorating qi, and promoting blood circulation (YQHX, *N* = 10), and the MI model + metoprolol (METO, *N* = 10). On day 2 after MI surgery, a dose of 8.2 g/kg/d YQHX and 5 mg/kg/d metoprolol (AstraZeneca Pharmaceutical Co., Ltd., National Drug Standard H32025391, Batch no. 1805A23) was administered. The same amount of water (distilled) was given to both groups of MI and sham operations. Allergic reactions were checked on days 3 and 7 after intragastric administration.

### 2.4. Echocardiogram

Before sampling, echocardiography (Visual Sonic, Vevo770, Canada) was conducted to examine the rats. For this, an injection of pentobarbital sodium (1%) was used as anesthesia, with the chest skin of the rats being supine. At the time of ultrasound, a state of normal physiology was maintained. For each mouse, 3 consecutive cardiac cycles were considered. FS (left ventricular short-axis ratio), left ventricular EF (ejection fraction), LVIDd (left ventricular end-diastolic diameter), and LVIDs (left ventricular end-systolic diameter) were measured.

### 2.5. Staining with Hematoxylin and Eosin (HE)

The myocardium tissue was fixed, dehydrated, embedded, sliced (4 *μ*m thick), and stained with HE. Then, through gradient down ethanol, sections were dewaxed and dehydrated. Staining of nuclei was performed using hematoxylin, followed by differentiation in HCL ethanol (1%). Then, a solution of red ethanol (1%) was used, followed by dehydration using gradient ethanol. The sections were microscopically observed, and images were acquired for evaluation.

The article "Impact of Yiqi Huoxue Decoction on the Relationship between Remodeling of Cardiac Nerves and Macrophages after Myocardial Infarction in Rats" was retracted in 2023. Reasons: unreliable results or conclusions; concerns about the data; concerns about the peer review; concerns about the citations.

### 2.6. Immunohistochemical Analyses

After dewaxing, paraffin sections were positioned in a repair chamber containing ethylenediaminetetraacetic acid (EDTA) antigen extraction buffer (pH 8.0) for the extraction of antigen in a steamer. The slides, after being inserted in phosphate-buffered saline (PBS, pH 7.4), were rinsed three times, followed by shaking on a decolorizing shaker, each time for 5 min. Endogenous peroxidase was blocked, a circle was drawn, and serum was used to seal it. This was followed by the addition of a primary antibody to the slides after gently discarding the blocking solution, placed in a damp box, and incubated at 4°C overnight. Next, the slides were inserted in PBS (pH 7.4) on a decoloring shaker and rinsed three times, each for 5 min. The slices were allowed to dry slightly, and a secondary antibody specific for the primary antibody was poured dropwise into the circle for covering the tissue and incubated at ambient temperature for 60 min. Then, the tissue was rinsed and incubated in horseradish peroxidase (HRP). After rinsing, DAB (3, 3′-diaminobenzidine) staining was continued; for this, the solution of PBS was eliminated, and a fresh solution of DAB (50–200 *μ*L) was added to individual pieces for dyeing the nuclei.

### 2.7. Western Blotting

The tissue samples were homogenized with a 1 mL radioimmunoprecipitation assay (RIPA) lysis buffer. For the extraction of proteins, the samples were dissolved for 30 minutes on ice, and the obtained proteins were quantified by employing a bicinchoninic acid (BCA) protein assay kit. The total load protein was 40 *µ*g and 20 *µ*L. The target protein's molecular weight was detected by gel isolation with appropriate proportions, and then electrophoresis and electrical conversion were performed. The polyvinylidene difluoride (PVDF) membrane following electroporation was submerged in Tris Buffer Saline Tween20 (TBST) sealing solution containing 5% milk. Antibodies against GAP43 (AB75810, Abcam), NGF (ab52918, Abcam), Semaphorin3A (SEMA-3A, AB11370, Abcam), tyrosine hydroxylase (TH, AB112, Abcam), actin (AB8226, Abcam), CD68 (AM25212, Abcam), CD163 (Ab82422, Abcam), CD86 (GTX34569, GeneTex), TLR4 (Proteintech, 19811-1-AP), and NF-*κ*B antibody (Ab16502, Abcam) were added and kept overnight. Relative expressions of proteins were determined by grayscale scanning gel imaging and electrochemiluminescence.

The article "Impact of Yiqi Huoxue Decoction on the Relationship between Remodeling of Cardiac Nerves and Macrophages after Myocardial Infarction in Rats" was retracted in 2023. Reasons: unreliable results or conclusions; concerns about the data; concerns about the peer review; concerns about the citations.

### 2.8. Statistical Analysis

All data were processed by SPSS22.0 software. The comparisons between multiple groups were in accordance with normal distribution, and a one-way assessment of variance was employed. If the variance was uniform, multiple comparisons between multiple groups were analyzed by least significant difference (LSD) to test the level. If the variance was uneven, Games–Howell is used for analysis. If the normal distribution was not met, nonparametric *k* independent samples were tested and *P* < 0.05 was deemed significant considering statistical standards.

## 3. Results

### 3.1. Alterations in Cardiac Function and Structure in MI Rats

Echocardiography is an effective and common technique to assess changes in cardiac activity. As shown in Figure 1(a), there was a significant decrease in EF and FS of rats in the MI group, an increase in LVIDs, and severely impaired cardiac function 3 and 7 days after MI. At 7 days, YQHX and METO groups exhibited a higher EF than that in the MI group and lower LVIDs levels than that in the MI group. HE staining is one of the common and intuitive methods for observing tissue morphology. HE staining showed (Figure 1(b)) that 3 days after MI, relative to the sham group, the MI group had structurally damaged and disordered myocardial cells with inflammatory cell infiltration. The pathological alterations in the YQHX intervention group were slightly fewer than those in the METO intervention group. Seven days after MI, the structure of myocardial cells in the group of sham was neat and occasionally broken. Regarding the MI group, the myocardial cell number at the edge of infarction decreased, the arrangement of myocardial tissue was disordered, and a large, remarkably high number of inflammatory cells were observed in the interstitium. In comparison to the MI group, myocardial cells in the YQHX intervention group were arranged continuously and neatly, and inflammatory infiltration of the extracellular interstitium was reduced. The pathological changes of the METO intervention group were similar to those of the Y group. In conclusion, YQHX can cause improvement in cardiac function after MI in rats and also decrease the impairment at the infarction area edge.

### 3.2. Function of YQHX on Factors for Nerve Remodeling in the Marginal Area of MI Rats

The study of NORI by Wang et al. [22] on MI rats showed that most of the regenerated nerve fibers were positive for TH, indicating that the regenerated nerve was mainly a mature sympathetic nerve. TH is a sympathetic nerve-specific marker, extensively distributed in the cytoplasm of norepinephrine nerve axons. It takes part in catecholamine synthesis, being a ring-ring-speed enzyme of catecholamine synthesis with remarkable specificity [24], and its positive detection can depict the sympathetic nerve distribution. The increase in nerve fibers leads to the increase in catecholamine release and the increase in sympathetic nerve activity, which is unbalanced with parasympathetic innervation. The positive distribution of TH in myocardia is associated closely with nerve remodeling after MI.

The article "Impact of Yiqi Huoxue Decoction on the Relationship between Remodeling of Cardiac Nerves and Macrophages after Myocardial Infarction in Rats" was retracted in 2023. Reasons: unreliable results or conclusions; concerns about the data; concerns about the peer review; concerns about the citations.

Immunohistochemical analyses in the MI marginal area showed (Figure 2(a)) that, 3 days after MI, there was a notable or complete reduction in the nerve fibers positive for TH in the sham group, with a uniform and consistent distribution among myocardial fibers in the direction of myocardial cells. In the MI group, nerve fibers positive for TH were increased significantly in density, coarse in shape, with random distribution. After treatment with METO and YQHX, the density and morphology distribution of nerve fibers positive for TH decreased relative to that in the MI group. The nerve growth factors, NGF and GAP43, can lead to uncontrolled regeneration and uneven density of cardiac nerves following MI. An inhibitor of nerve growth, SEMA-3A, impedes sympathetic overgrowth. As shown in Figure 2(b), on days 3 and 7, the expression of TH, NGF, and GAP43 in group *M* was higher at significant levels relative to those in group S, while SEMA-3A expression was low. On days 3 and 7, the expression of TH, GAP43, and NGF in the YQHX group and the METO group decreased relative to that in group *M*. At day 7, both YQHX and METO upregulated SEMA-3A expression. Therefore, after METO and YQHX intervention, TH, GAP43, and NGF expressions were downregulated, and SEMA-3A expression could be upregulated 7 days later as shown in Figure 2(c).

### 3.3. Effects of YQHX on Macrophages and Inflammation-Related Proteins in the Marginal Area of Myocardial Infarction Rats

Macrophages are differentiated mainly into two subtypes after activation [25]: the classical activated macrophage M1 and the selective activated macrophage M2 subtypes. Molecular markers on the surface of macrophages are also an important basis for the classification of macrophages. CD68 and CD86 are the second surface markers of M-type macrophages, which can secrete inflammatory factors like tumor necrosis factor (TNF)-*α*, interleukin (IL)-1, and IL-6 after activation. Activation of M2-type macrophages increases the expression of CD68 and CD163 and secretion of transforming growth factor-*β* (TGF-*β*), IL-10, IL-4, and other anti-inflammatory factors [26, 27]. Toll-like receptors (TLR), mainly distributed on the surface of immune cells, for instance, mononuclear macrophages, lymphocytes, and dendritic cells, are also expressed in the heart and are considered a bridge between immune response and inflammatory response [28, 29]. Nuclear factor kappa B (NF-*κ*B) is an essential regulating factor for the transcription of inflammatory genes and is essential for the macrophage inflammatory response. After activation, NF-*κ*B is transferred from the cytoplasm into the nucleus and is essential for regulating inflammatory factors [30]. The activated macrophage surface TLR4 receptor is activated and binds to the corresponding ligand to activate NF-*κ*B.

The article "Impact of Yiqi Huoxue Decoction on the Relationship between Remodeling of Cardiac Nerves and Macrophages after Myocardial Infarction in Rats" was retracted in 2023. Reasons: unreliable results or conclusions; concerns about the data; concerns about the peer review; concerns about the citations.

According to Figure 3(a), relative to the sham group, other groups had significantly increased CD86 on day 3 and decreased in group YQHX and METO in comparison to the group of MI on day 7 (Figure 3(b)). The change of CD163 was not obvious at 3 days (Figure 3(c)) but increased at 7 days (Figure 3(d)).

Western blot results showed (Figure 4) that, on day 3, CD86 content underwent an increase in the model group and enhanced in the MI group on day 7. In comparison with the group of MI, the protein content of CD163 in the myocardial tissue at the edge of infarction in the medication group had a substantial increment. In addition, the CD163 expression in the medication group increased significantly on the 7th day compared to that on the 3rd day. On day 3 after MI, a significantly higher expression of TLR4 and NF*κ*B was detected in the group of MI than in the group of sham, but the change was not obvious in the medication group. On day 7 after MI, TLR4 and NF-*κ*B expressions were lower in the medication group than in the MI group.

According to the above results, M1-type CD86 macrophages promoting inflammation increased significantly on day 3 after MI. On day 7, macrophages of M2-type CD163, which inhibits inflammation, increased, consistent with the differentiation process of macrophages after inflammation. It is noteworthy that, after 7 days of continuous administration, CD86 expression in the medication group decreased relative to that in the model group, while the content of CD163 increased superior to that in the model group. Concurrently, the levels of inflammatory factors TRL4 and NF*κ*B also decreased. Combined with immunohistochemical findings, further clarification proves that YQHX can promote M2-type macrophage secretion and decrease Ml breakdown cell to minimize MI in the rat with myocardial inflammatory response in the edge area of infarction to reduce the myocardial injury, promote the freshmen, reshape myocardial tissue, and improve heart function and recovery.

## 4. Discussion

In this study, we examined the mechanism by which YQHX inhibits MI-induced sympathetic nerve regeneration. Sympathetic nerve remodeling after MI may result in arrhythmias and sudden death. YQHX downregulates the expression of TLR4 and NF*κ*B in MI rats, induces macrophage phenotype transformation from M1 to M2, and reduces the expression of nerve growth factors, thus improving sympathetic nerve germination and innervation, consistent with previous findings. TH-positive nerve fiber clusters were found at the edge of MI, and YQHX treatment improved sympathetic remodeling by decreasing TH-positive nerve fiber density, decreasing NGF and GAP43 expression, and increasing SEMA-3A expression.

The article "Impact of Yiqi Huoxue Decoction on the Relationship between Remodeling of Cardiac Nerves and Macrophages after Myocardial Infarction in Rats" was retracted in 2023. Reasons: unreliable results or conclusions; concerns about the data; concerns about the peer review; concerns about the citations.

The pathogenesis of MI is closely associated with the acute inflammatory response. The inflammatory response due to MI aggravates tissue damage and functional impairment, and the inflammatory response is also the prerequisite for healing and tissue scar formation. Anti-inflammatory therapy can reduce the scope of infarction in treating MI to prevent cardiac remodeling and further cardiac failure [31]. At the same time, sympathetic nerve germination after MI is closely related to inflammatory processes [8, 9, 32, 33] that lead to NGF synthesis locally by inflammatory cells, including myofibroblasts and macrophages. Nerve growth factor (NGF) is a powerful neurochemokine that is essential for sympathetic nerve germination, survival, differentiation, and synaptic functions during heart injury [34]. Studies have shown that direct intracardial transduction lentivirus vectors carry NGF-targeted siRNA (short interfering RNA) to downregulate NGF. It can significantly improve the remodeling and budding of the sympathetic nerve [35]. Moreover, Hasan et al. [13] opined that NGF is a necessary condition for the germination of the sympathetic nerve, and NGF is widely expressed in the area around infarction and is associated with the aggregation of a large number of filtered macrophages and myofibroblasts. Wernli et al. [12] confirmed that macrophage consumption after MI significantly reduced NGF content and inhibited sympathetic overregulation.

As reported in previous studies, this study data also showed that after MI, NGF, and GAP-43 expressions were upregulated, SEMA-3A expressions were downregulated, TH-positive nerve fiber density was increased, and sympathetic overinnervation selectively occurred in regions containing a large number of macrophages. YQHX downregulates NGF expression by inhibiting the differentiation of macrophages; therefore, it is like that macrophages may be involved in the relationship between inflammation and cardiac sympathetic innervation induced by MI through the regulation of NGF expression.

The article "Impact of Yiqi Huoxue Decoction on the Relationship between Remodeling of Cardiac Nerves and Macrophages after Myocardial Infarction in Rats" was retracted in 2023. Reasons: unreliable results or conclusions; concerns about the data; concerns about the peer review; concerns about the citations.

At the early stage of 1–3 days after myocardial infarction, M1-type macrophages mainly secreted TNF-*α*, inducible nitric oxide synthase (iNOS), IL-6, and additional factors involved in inflammation response, which mainly phagocytosed apoptotic and necrotic cell fragments. However, long-term inflammatory reactions lead to poor ventricular remodeling. From 3 to 7 days (middle and late stage), M2 macrophages are the primary type, and type 2 predominantly secretes arg-1, TGF-*β*, etc., which mainly promote angiogenesis and degradation of extracellular matrix, stimulate fibroblasts into myofibroblast differentiation, participate in the occurrence of myocardial fibrosis [36, 37], and participate in anti-inflammatory and tissue repair [38,39]. CD68 macrophages and *α* fibroblasts are important sources of NGF synthesis and release. In MI rat models, clodronate liposomes can reduce the density of sympathetic axons and NGF expression by 69% without affecting the number of T cells; hence, macrophages are considered the main cause of sympathetic nerve regeneration after MI [12, 13]. The activation of P2X purinoceptor 7 (P2X7R) of M1-type macrophages promotes the generation of NLR family pyrin domain containing 3 (NLRP3)/IL-1*β*, increases the generation of NGF, and causes the pathological process of sympathetic nerve regeneration after MI [40]. Blocking P2X7R can inhibit NLRP3/IL-1*β* pathway and reduce sympathetic nerve regeneration after MI. Therefore, it is speculated that M1-type macrophages of the heart promote the formation of NGF, participate in cardiac nerve remodeling, and impact arrhythmia after MI, concurrent with the results of this study.

Herein, the infiltration of M1 and M2 macrophages in the injured myocardial tissue was observed by immunohistochemical and western blotting. CD86 macrophages were more infiltrated in the myocardial tissue after MI. Further analysis was made on the classification of infiltrated macrophages. A decrease in inflammatory cells was observed. Compared with the MI group, the inflammatory M1-type CD86 macrophages decreased, while the anti-inflammatory M2-type CD163-positive macrophages increased significantly, thus indicating that YQHX can alleviate myocardial inflammation in the infarct margin of MI rats by promoting the secretion of M2-type macrophages and inhibiting the secretion of M1-type macrophages to alleviate myocardial injury, promote the regeneration and remodeling of myocardial tissue, and facilitate the recovery of cardiac function.

This study suggests that YQHX can affect the phenotypic changes of macrophages after MI, which may downregulate NGF expression. YQHX was confirmed to polarize macrophages into the M2 phenotype, and the levels of TLR4 and NFKB are downregulated. Meanwhile, GAP-43 and NGF expressions and the TH and positive nerve fibers density also decreased, and the expression of SEMA-3A increased. Thus, we hypothesize that the phenotype of macrophages is important for sympathetic regeneration.

The article "Impact of Yiqi Huoxue Decoction on the Relationship between Remodeling of Cardiac Nerves and Macrophages after Myocardial Infarction in Rats" was retracted in 2023. Reasons: unreliable results or conclusions; concerns about the data; concerns about the peer review; concerns about the citations.

## 5. Conclusion

In summary, through these experimental results, we confirm that YQHX can affect the phenotypic changes of macrophages after MI and regulate the expression of neuro-associated factors after MI. It is speculated that the phenotype of macrophages is essential for sympathetic nerve regeneration, and YQHX has an effect on sympathetic nerve regeneration. However, the regulatory mechanisms of YQHX with macrophages and sympathetic nerves should be studied further in cellular and animal experiments. With the deepening of the investigation on sympathetic nerves and inflammation after MI, the early intervention of inflammation and factors associated with nerve remodeling and the application of traditional Chinese medicine in the convalescence stage of MI may be a significant target and therapy plan to diminish and treat cardiovascular diseases in the next years.

## Figures and Tables

**Figure 1:** (a) Cardiac function and echocardiogram of rats in each group after days 3 and 7 of MI (myocardial infarction) (*N* = 9). ^##^*P* < 0.01, vs. the sham operation group; ^*∗*^*P* < 0.01, vs. the MI model group. (b) Histopathological staining using hematoxylin and eosin of the tissue in the infarct marginal area of rats with MI in each group (scale bar = 200 *μ*m).

**Figure 2:** (a) Immunohistochemical staining for examining the positive, sympathetic nerve fibers at the edge of MI (myocardial infarction) in rats 3 days after MI (scale). (b) Immunohistochemical staining was used to observe the positive, sympathetic nerve fibers at the edge of myocardial infarction in rats 7 days after MI (myocardial infarction). (c) The influence of YQHX on GAP43, TH, SEMA-3A, and NGF expression. ^##^*P* < 0.01, vs. the sham operation group; ^*∗*^*P* < 0.01, vs. MI.

**Figure 3:** (a) Immunohistochemical analysis to detect the CD86 macrophages at the edge of myocardial infarction (MI) in rats 3 days after myocardial infarction. (b) Immunohistochemical analysis to observe the CD86 macrophages at the edge of MI in rats 7 days after myocardial infarction. (c) Immunohistochemical analysis to observe the CD163 macrophages at the edge of MI in rats 3 days following myocardial infarction. (d) Immunohistochemical analysis to observe the CD163 macrophages at the edge of MI in rats 7 days after myocardial infarction.

**Figure 4:** The expression of CD86, CD163, TLR4, and NF*κ*B in each group of rats; the tissue of the infarct marginal area was examined. ^##^*P* < 0.01, vs. the sham operation group; ^*∗*^*P* < 0.01, vs. the MI model group; a*P* < 0.01, vs. the model group of 3 days.

The article "Impact of Yiqi Huoxue Decoction on the Relationship between Remodeling of Cardiac Nerves and Macrophages after Myocardial Infarction in Rats" was retracted in 2023. Reasons: unreliable results or conclusions; concerns about the data; concerns about the peer review; concerns about the citations.

## Data Availability

The data employed to support the achievements of the present survey can be obtained from the corresponding author upon request.

## Abbreviations

MI: Myocardial infarction
YQHX: Yiqi Huoxue decoction
TLR4: Toll-like receptor 4
NF-*κ*B: Nuclear factor kappa B
GAP43: Growth-associated protein 43
NGF: Nerve growth factor
TH: Tyrosine hydroxylase
TCM: Traditional Chinese medicine
HPLC-LTQ-Orbitrap MS: The high-performance liquid chromatography coupled with linear ion trap quadrupole Orbitrap high-resolution mass spectrometry
API: Active pharmaceutical ingredients
SPF: Specific pathogen free
LAD: Left anterior descending
ECG: Electrocardiogram
METO: Metoprolol
EF: Ejection fraction
LVIDd: Left ventricular end-diastolic diameter
LVIDs: Left ventricular end-systolic diameter
HE: Hematoxylin and eosin
EDTA: Ethylenediaminetetraacetic acid
PBS: Phosphate buffered saline
HRP: Horseradish peroxidase
DAB: 3, 3′-diaminobenzidine
PVDF: Polyvinylidene difluoride
TBST: Tris buffer saline tween20
TNF: Tumor necrosis factor
IL: Interleukin
TGF-*β*: Transforming growth factor-*β* definition
iNOS: Inducible nitric oxide synthase
siRNA: Short interfering RNA
SEMA-3A: Semaphorin3A
NLRP3: NLR family pyrin domain containing 3
P2X7R: P2X purinoceptor 7
LSD: Least significant difference
BCA: Bicinchoninic acid
RIPA: Radioimmunoprecipitation assay.
